# Nanosilver Dressing in Treating Deep II Degree Burn Wound Infection in Patients with Clinical Studies

**DOI:** 10.1155/2021/3171547

**Published:** 2021-12-13

**Authors:** Bin'e Wu, Fengchun Zhang, Wenbin Jiang, Aiyan Zhao

**Affiliations:** Department of Disinfection and Supply, Weifang People's Hospital, Weifang, China

## Abstract

**Background:**

Patients' clinical antibiotic treatment of deep II degree burns usually fails to achieve the ideal effect; in order to avoid the late result in pigmentation, scarring, and even limb dysfunction, it also needs to deal effectively with burn wounds.

**Aim:**

The purpose of this study is to evaluate nanosilver dressing in treating deep II degree burn wound infection in patients with clinical studies.

**Materials and Methods:**

106 burn patients were classified into the Sulfadiazine Silver Cream (SSC) group (*n* = 53) and the Nanosilver Burn Dressing (NSBD) group (*n* = 53). Both of them received basic wound treatment, and wound healing time and pigmentation fading away time of all patients were recorded. And the wound healing rate of the patients was calculated. Serum levels of tumor necrosis factor alpha (TNF-*α*) and interleukin-1beta (IL-1*β*) were detected pre- and posttreatment.

**Results:**

After basic treatment for all patients, Sulfadiazine Silver Cream was used in the SSC group, and Nanosilver Burn Dressing was used in the NSBD group. It was observed that after treatment, compared with the SSC group, there was significant efficiency; wound healing rate, healing time, and pigmentation fading away time were shortened in the NSBD group, and IL-1*β* levels were decreased, and the positive rate of bacterial culture was decreased (all *P* < 0.05).

**Conclusion:**

Nanosilver Burn Dressing in treating deep II degree burns can effectively reduce the wound infection and promote wound healing. The curative effect was distinct, which was worthy of popularization and application.

## 1. Introduction

Burn is a kind of tissue damage caused by fire, electricity, high temperature, and strongly hot objects or chemicals. Clinically, according to the depth and scope of the injured tissue in patients, it is from deep to shallow divided into III, II, and I degrees [1]. The II degree burn injury is characterized by skin growing white or red at the bottom of the blister. The blisters are filled with a clear and viscous fluid that turns white when pressed and is painful [2]. A burn that involves the dermis but retains the dermis residue is a deep II degree burn wound [3]. Due to the deep II degree burns of deep burn wounds and wide range, it is often easy to cause wound infection [2]. Studies have shown that wound infection leads to prolonged hospital stay, which will increase medical costs and, in severe cases, can cause sepsis, multiple organ failure, and even death [4]. In general, antibacterial therapy alone cannot achieve satisfactory efficacy and prognosis, and wound management has a great influence on the prognosis. Improper wound treatment can also lead to pigmentation, growth of scar, and even limb dysfunction. Therefore, effective treatment of burn wounds, especially to avoid wound infection, is of great significance for the recovery of prognosis. Sulfadiazine Silver Cream is a commonly used sulfadiazine antimicrobial agent. Although it can achieve good antimicrobial effect, its irritation is relatively large and it is easy to cause scarred burn wounds in patients [5]. Nanosilver Burn Dressing contains nanoscale (most of the diameter is 25 nm) elemental silver, which slowly releases silver ions. On the one hand, silver ions bind to bacterial bases and inhibit DNA replication; on the other hand, silver ion proteins interact with bacterial proteins to generate silver proteins and inactivate bacteria. Other studies have shown that nanosilver dressing not only has anti-inflammatory effect but also can promote wound healing [6]. And at present, the application of silver nanoparticles in deep II degree burn wound infection in patients is very little. So, this study applied Sulfadiazine Silver Cream as a control, aimed at exploring influence of Nanosilver Burn Dressing on patients with II degree burn wound infection and observing wound healing. We present the result reports as follows.

## 2. Materials and Methods

### 2.1. Materials

After approval by the Medical Ethics Committee, the subjects of this study were burn patients admitted to our hospital from March 2016 to March 2020. Inclusion criteria include the following: (1) in accordance with the “four-point method,” on admission diagnosis of deep II degree burns [7]; (2) treatment within 36 hours after burn; (3) no severe shock; (4) no metabolic diseases; (5) no other complicated injuries or serious infections; and (6) informed consent of family members. Exclusion criteria include the following: (1) severe inhalation injury; (2) consciousness disorder; (3) lesions of the heart, liver, kidney, and other important organs; (4) tumor; (5) have blood system diseases; and (6) women who are pregnant or lactating. A total of 106 cases were selected and classified into the SSC group (*n* = 53) and the NSBD group (*n* = 53) in line with the random number table method. There were no significant differences between the SSC group and the NSBD group in gender, burn reason, burn site, age, and burn area level (*P* > 0.05), and there was comparability between the two groups (Table 1, Figures 1 and 2).

### 2.2. Materials and Methods

#### 2.2.1. Basic Wound Treatment

After admission, blood pressure, pulse, and electrocardiogram of all patients were monitored. Oxygen inhalation, calm, and volume expansion therapy were given according to the actual condition. Fluid supplementation was given to correct water and electrolyte disturbance and anti-infection in a timely manner. The burn wound was washed with 0.9% sodium chloride solution and disinfected with iodine volt. Necrotic skin was removed from the wound, and the blisters were drained if necessary.

#### 2.2.2. Wound Dressing

The SSC group used Sulfadiazine Silver Cream (production enterprises: Kunming Flame Pharmaceutical (Group) Co., Ltd., approval number: GUOYAOZHUNZI H20057720, specification: 1% 500 g) treatment. The NSBD group used Nanosilver Burn Dressing (manufacturing enterprises: Anxin Nano Biotech (Zhuhai) Co., Ltd., approval number: GUOJIEZHUZHU 20163640177, specifications: 10 × 15 cm, 20 × 20 cm, and 35 × 40 cm) treatment (Figure 3). The wounds of patients in both groups were regularly cleaned and bandaged for dressing change once every 2 d. Each time, the residual drugs on the wound were removed before dressing change, and finally, the wound was bandaged with sterile gauze. The dressings were changed continuously and would not be stopped until the patients' wound healed.

### 2.3. Observation Target

#### 2.3.1. Efficacy

After 14 days of treatment, the patients were evaluated, including inefficiency, effectivity, significant effectivity, and recovery. The ineffective ones have no improvement or even aggravation of the wound surface after dressing change or subcutaneous purulent infection. For effectivity, the wound surface was basically free of infection and the pain was relieved after dressing change. After dressing change, the wound surface was significantly improved, the pain was largely relieved, and the bleeding and exudate were quickly absorbed. For recovery, the wound was improved without infection, the pain was significantly relieved, and the bleeding and exudate were rapidly absorbed. Total significant effectivity = (significant effectivity + recovery) cases/total cases × 100% [8].

#### 2.3.2. Wound Prognosis Speed

Wound healing time and pigmentation fading away time of all patients were recorded. For wound healing, on the 7th, 14th, and 28th days of treatment, the wound healing rate of the patients was calculated. The wound healing rate is the burn wound area minus the unhealed wound area divided by the percentage of the burn wound area.

#### 2.3.3. Inflammation

Serum levels of tumor necrosis factor alpha (TNF-*α*) and interleukin-1beta (IL-1*β*) were detected pre- and posttreatment. For methods, peripheral blood was collected and centrifuged, and the supernatant was retained and stored in a frozen environment. Serum TNF-*α* and IL-1*β* were examined by an enzyme-linked immunosorbent assay. For bacterial culture results, after 14 days of treatment, the wound secretions of all patients were bacteriologically cultured, and bacterial species were identified, and the bacterial culture results were analyzed to calculate the positive rate of the two groups [3].

### 2.4. Statistical Analysis

The data was input and analyzed in SPSS17.0 software. The measurement data conforming to normal distribution was expressed as the mean ± standard deviation (SD), after performing the *t*-test. Counting data was expressed as percentage, and the chi-squared test was carried out. *P* < 0.05 indicated a statistically significant difference.

## 3. Results and Discussion

### 3.1. Comparison of Total Effective Rate, Prognosis Rate, and Wound Healing Rate

Compared with the 60.38% of the SSC group, the total significant effectivity 81.13% of the NSBD group was significantly higher (Table 2, Figure 4). Compared with the SSC group, the healing time and pigmentation fading away time in the NSBD group were significantly shorter (Table 3, Figure 5). And the wound healing rate was significantly higher on the 7th, 14th, and 28th days of treatment (Table 4, Figure 6). All above comparisons were *P* < 0.05.

### 3.2. TNF-*α*, IL-1*β*, and Positive Rate

TNF-*α* and IL-1*β* levels decreased in both groups after treatment, and those of the NSBD group was significantly lower (*P* < 0.05) (Table 5, Figure 7). Compared to the SSC group, the positive rate of the NSBD group was significantly lower (18.87% vs. 30.19%, *P* < 0.05). Compared with the 30.19% of the SSC group, the positive rate 18.87% of the NSBD group was significantly lower (Table 6, Figure 8).

### 3.3. Discussion

Deep II degree burns belong to severe burns and have a wide range from burns, the wound healing is slow, and the burn injury is to the dermis, which can lead to large scars to patients. According to data shown, giving deep II degree burn wounds of patients effective treatment to promote the wound healing and pigmentation fade, to reduce infection, and to improve the curative effect has positive significance [1]. Although Sulfadiazine Silver Cream can kill fungi, Gram-negative bacteria, and Gram-positive bacteria, it is very easy to cause local microcirculation blockage of patients, which is not conducive to the prognosis of burn wounds, and even aggravate the condition [9]. So, exploring the application effect of Nanosilver Burn Dressing on deep II degree burns is of great importance.

The results of this study indicated that in comparison with the patients who used Sulfadiazine Silver Cream for dressing change, the total significant effectivity and wound healing rate of the patients who used Nanosilver Burn Dressing were significantly higher, and the positive rate of wound secretion was significantly reduced after bacterial culture. If wound infection is caused by improper treatment of burn wounds, serious complications such as blood poisoning, septicopyemia, and multiple organ failure may occur in patients, which will increase the difficulty of treatment [10]. Bacterial culture is the “gold standard” for judging bacterial infection, and the decrease of the positive rate of bacterial culture in wound secretions is conducive to the recovery of the prognosis of burn wounds [11]. The bactericidal mechanism of nanoscale silver ions contained in the Nanosilver Burn Dressing is that they penetrate the cytoplasm of bacteria to block the synthesis of respiratory enzymes and kill them [12]. In addition, silver ions released slowly by the Nanosilver Burn Dressing after meeting water act on the burn wound and have a longer bactericidal effect. The particle size of silver ions is small, and the specific surface area is large, which enables its surface to fully contact with the burn wound, thus achieving effective sterilization effect. Nanosilver has the characteristics of strong bactericidal effect, wide antibacterial spectrum, and no drug resistance. It has the killing effect on the main bacteria infecting patients' burn wounds, such as Staphylococcus aureus, Pseudomonas aeruginosa, Escherichia coli, Acinetobacter baumannii, and Staphylococcus epidermidis. This reduces the positive rate of bacterial culture results, reduces the probability of wound infection, facilitates effective wound healing, increases the wound healing rate, and significantly improves the curative effect [13, 14]. Nanosilver Burn Dressing significantly shortened the healing time and pigmentation fading away time. Studies have shown that the activity of nanosize silver particles is very strong and able to activate and promote tissue growth and repair tissue damage. It can produce biological heat effect to improve blood circulation of the burn tissue around, which gives skin cells and dermis fibroblasts rapid growth and keeps the connective tissue fresh to replenish the damaged tissue [15]. Finally, on the one hand, wound healing will be accelerated; on the other hand, the pigmentation will be replaced by new tissue continuously, and finally, pigmentation will disappear quickly and scar growth will be reduced. The results also showed that TNF-*α* and IL-1*β* levels were significantly reduced in the object of study treated with Nanosilver Burn Dressing, indicating a mild inflammatory response in the patients. Both TNF-*α* and IL-1*β* are proinflammatory cytokines, which are low expressed in a normal human body, but their levels are abnormally elevated in the process of inflammatory response. Therefore, TNF-*α* and IL-1*β* can reflect the inflammatory situation in burn patients.

Studies have shown that TNF-*α* is secreted by activated macrophages, which promotes the adhesion, migration, and infiltration of inflammatory cells, and ultimately leads to the intensification of the inflammatory response of monocyte macrophages [16]. IL-1*β* mainly secreted by monocytes, fibroblasts, and endothelial cells can cause T cells to release large amounts of interleukin-2 through the activation of platelet growth factor and colony-stimulating factor and participate in the body's immune response [17].

However, researches on nanosilver dressing need further expansion. For instance, future studies could examine the optimal effects on the human body. Structure alteration could be performed in nanosilver dressing to obtain efficiency and a substitute for chemical synthetic nanosilver particles. To sum up, dressing change with Nanosilver Burn Dressing can effectively reduce the inflammatory response of the body and reduce the inflammation caused by infection in burn patients, thus having an anti-inflammatory effect. It can be proved that nanosilver dressings have an optimistic potential in wound infection healing. Appropriate utilization and development of nanosilver materials combined with continued research can improve the performance of nanosilver in terms of its physical, chemical, and biological aspects, thereby providing better medical conditions to patients.

## 4. Conclusion

Deep II degree burn wounds damage more seriously; improper handling can cause serious complications and even death. Even if no infection occurs in patients during conventional treatment, the pigmentation produced after wound healing is difficult to subside, and eventually, scarring is often left. Therefore, it is very important to prevent and cure wound infection in burn patients. In Nanosilver Burn Dressing, the nanosized (25 nm) silver elomer is attached to the surface of the cotton fiber and is slowly released after being applied to the burn wound. Then, the silver elomer is combined with the negatively charged bacterial protein to make it denatured, crack, and die to achieve the purpose of sterilization finally. Therefore, when Nanosilver Burn Dressing is applied in the process of burn wounds, it can enter deep tissue to kill bacteria, reduce inflammation, promote wound healing, and inhibit scar growth, with significant effect and high clinical application value.

## Figures and Tables

**Figure 1:** The general information: (a) gender; (b) burn reason; (c) burn site. Comparison of gender, burn cause, and burn site between the two groups, *P* > 0.05. Sulfadiazine Silver Cream (SSC) group (*n* = 53) and Nanosilver Burn Dressing (NSBD) group.

**Figure 2:** The age and fire burn TBSA: (a) age; (b) fire burn TBSA. Compared the two groups' age and fire burn TBSA, *P* > 0.05. TBSA: total body surface area. Sulfadiazine Silver Cream (SSC) group (*n* = 53) and Nanosilver Burn Dressing (NSBD) group.

**Figure 3:** Nanosilver. Nanosilver particle size is nanoscale (mostly 25 nm) metallic silver eleles, which have a strong inhibition and killing effect on pathogenic microorganisms. And there is no drug resistance.

**Figure 4:** Evaluation of treatment efficacy of NSBD. The significant efficiency of the NSBD group was higher, *P* < 0.05. Sulfadiazine Silver Cream (SSC) group (*n* = 53) and Nanosilver Burn Dressing (NSBD) group.

**Figure 5:** To compare prognosis of speed. The healing time and pigmentation fading away time of the NSBD group were shortened, *P* < 0.05. Sulfadiazine Silver Cream (SSC) group (*n* = 53) and Nanosilver Burn Dressing (NSBD) group.

**Figure 6:** Wound healing rate analysis. The wound healing rate of the NSBD group on the 7th, 14th, and 28th days of treatment was higher, *P* < 0.05. Sulfadiazine Silver Cream (SSC) group (*n* = 53) and Nanosilver Burn Dressing (NSBD) group.

**Figure 7:** Determination of TNF-*α* and IL-1*β* levels. (a) Prior to treatment; (b) posttreatment. After treatment, both groups' TNF-*α* and IL-1*β* levels were decreased, and the NSBD group was lower, *P* < 0.05. Sulfadiazine Silver Cream (SSC) group (*n* = 53) and Nanosilver Burn Dressing (NSBD) group.

**Figure 8:** To determine positive rate after NSBD treatment. The NSBD group's positive rate was lower, *P* < 0.05. Sulfadiazine Silver Cream (SSC) group (*n* = 53) and Nanosilver Burn Dressing (NSBD) group.

**Table 1:** The general information.

Group	Gender (case)		Age ($\bar{x}\pm s$, year)	Fire burn TB SA ($\bar{x}\pm s$, %)	Burn reason (case)		Burn site (case)		
	Male	Female			*Brulure de flamme*	Hot liquid scald	Head-face-neck	Body	Arms and legs
SSC group (*n* = 53)	31 (58.49%)	22 (41.51%)	40.26 ± 4.12	20.34 ± 1.68	28 (52.83%)	25 (47.17%)	21 (39.62%)	19 (35.85%)	13 (24.53%)
NSBD group (*n* = 53)	38 (71.70%)	15 (28.30%)	41.03 ± 3.51	20.55 ± 2.06	30 (56.60%)	23 (43.40%)	17 (32.08%)	20 (37.74%)	16 (30.19%)
*χ* ^2^/*t*/*Z*	2.034		1.036	0.575	0.152		-0.860		
*P*	0.154		0.303	0.566	0.696		0.390		

Note. SSC: Sulfadiazine Silver Cream; NSBD: Nanosilver Burn Dressing; TBSA: total body surface area.

**Table 2:** Efficacy.

Group	Inefficiency	Effectivity	Significant effectivity	Recovery	Significant effectivity rate
SSC group (*n* = 53)	2 (3.77%)	19 (35.85%)	14 (26.42%)	18 (33.96%)	32 (60.38%)
NSBD group (*n* = 53)	0	10 (18.87%)	15 (28.30%)	28 (52.83%)	43 (81.13%)
*t*					5.517
*P*					0.019

Note. SSC: Sulfadiazine Silver Cream; NSBD: Nanosilver Burn Dressing.

**Table 3:** Prognosis of speed $\left(\bar{x}\pm s\right).$

Group	Healing time (d)	Pigmentation fading away time (d)
SSC group (*n* = 53)	23.21 ± 3.52	75.21 ± 5.34
NSBD group (*n* = 53)	17.37 ± 4.06	41.42 ± 7.19
*t*	7.912	27.470
*P*	<0.001	<0.001

Note. SSC: Sulfadiazine Silver Cream; NSBD: Nanosilver Burn Dressing.

**Table 4:** Wound healing rate $\left(\bar{x}\pm s,\%\right)$.

Time of therapy	SSC group (*n* = 53)	NSBD group (*n* = 53)	*t*	*P*
The 7th day	35.67 ± 3.98	42.15 ± 4.02	8.339	<0.001
The 14th day	72.36 ± 11.64	85.36 ± 12.31	5.586	<0.001
The 28th day	88.92 ± 6.68	96.37 ± 7.21	5.518	<0.001

Note. SSC: Sulfadiazine Silver Cream; NSBD: Nanosilver Burn Dressing.

**Table 5:** TNF-*α* and IL-1*β*$\left(\bar{x}\pm s\right)$.

Group	TNF-*α* (ng/L)		IL-1*β* (ng/L)	
	Prior to treatment	Posttreatment	Prior to treatment	Posttreatment
SSC group (*n* = 53)	193.14 ± 25.17	177.13 ± 18.22^∗^	238.25 ± 35.16	149.14 ± 30.28^∗^
NSBD group (*n* = 53)	192.85 ± 25.41	154.39 ± 17.63^∗^	235.69 ± 38.26	126.27 ± 18.94^∗^
*t*	0.059	6.530	0.359	4.662
*P*	0.953	<0.001	0.721	<0.001

Note. ^∗^Compared with the same group prior to treatment, *P* < 0.05. SSC: Sulfadiazine Silver Cream; NSBD: Nanosilver Burn Dressing; TNF: tumor necrosis factor; IL: interleukin.

**Table 6:** Positive rate.

Group	Staphylococcus epidermidis	Acinetobacter baumannii	Staphylococcus aureus	Escherichia coli	Pseudomonas aeruginosa	Positive rate
SSC group (*n* = 53)	2 (3.77%)	3 (5.66%)	4 (7.55%)	5 (9.43%)	2 (3.77%)	16 (30.19%)
NSBD group (*n* = 53)	2 (3.77%)	2 (3.77%)	2 (3.77%)	1 (1.89%)	3 (5.66%)	10 (18.87%)
*t*						1.835
*P*						0.176

Note. SSC: Sulfadiazine Silver Cream; NSBD: Nanosilver Burn Dressing.

## Data Availability

If any qualified researcher needs, all the raw data could be accessed by contacting the corresponding author.
